# RDFNet: A Fast Caries Detection Method Incorporating Transformer Mechanism

**DOI:** 10.1155/2021/9773917

**Published:** 2021-11-10

**Authors:** Hao Jiang, Peiliang Zhang, Chao Che, Bo Jin

**Affiliations:** ^1^Key Laboratory of Advanced Design and Intelligent Computing (Dalian University), Ministry of Education, Dalian 116622, China; ^2^School of Innovation and Entrepreneurship, Dalian University of Technology, Dalian 116024, China

## Abstract

Dental caries is a prevalent disease of the human oral cavity. Given the lack of research on digital images for caries detection, we construct a caries detection dataset based on the caries images annotated by professional dentists and propose RDFNet, a fast caries detection method for the requirement of detecting caries on portable devices. The method incorporates the transformer mechanism in the backbone network for feature extraction, which improves the accuracy of caries detection and uses the FReLU activation function for activating visual-spatial information to improve the speed of caries detection. The experimental results on the image dataset constructed in this study show that the accuracy and speed of the method for caries detection are improved compared with the existing methods, achieving a good balance in accuracy and speed of caries detection, which can be applied to smart portable devices to facilitate human dental health management.

## 1. Introduction

Dental caries is a prevalent disease of the human oral cavity that has a great impact on human quality of life. Data from the National Health and Nutrition Examination Survey, 2011–2012, showed that among children aged 2–8 years, 37% had dental caries in their primary teeth. Among adolescents aged 12–19 years, the prevalence of dental caries in permanent teeth was 58%. Approximately 90% of adults aged ≥20 years had dental caries [1]. Therefore, the detection of dental caries can provide reliable clinical reference to doctors and effectively avoid the onset or the further severity of dental caries, which is of great significance to improving the quality of human life.

With the advances of deep-learning methods in computer vision, many such methods have been applied to caries detection to improve the accuracy of detection and relieve the dentists' workload. For example, Suryani et al. [2] used mask R-CNN to detect objects in dental panoramic X-ray images, which saved time and improved the quality of dentists' diagnoses by automatically detecting panoramic X-ray images. Majanga et al. [3] proposed a deep learning-based technique for dental caries detection named blob detection. The proposed technique automatically detects hidden and inaccessible dental caries lesions. The process of detection and classifying dental caries achieved the results of 97% and 96% for the precision and recall values, respectively. The above methods for caries detection are mainly based on X-ray images. However, the X-ray images must be captured and acquired by professional equipment and specialized technicians, which is expensive and cumbersome. It has become increasingly easy to acquire digital images due to the popularity of portable devices and the development of biological storage technology [4]. Caries detection becomes quicker and more convenient based on these digital images, making it possible to conduct detection anytime and anywhere. Therefore, the use of digital images for caries detection has become a new demand in human dental health management.

Saini et al. [5] used digital images of dental caries for early classification and prevention of dental caries. They used four convolutional neural networks including ResNet50, all of which achieved good classification accuracy. However, their study only classified the images of caries without detecting the type of caries and lesion area. To our knowledge, no study has been conducted on the detection of dental caries based on digital images, mainly because of the lack of large-scale digital image datasets of annotated dental caries. Caries detection is an object detection task, and the popular object detection algorithms are all supervised deep-learning methods, which require a large amount of annotated data to train the model. The caries images must be annotated by professional dentists, which is troublesome and laborious. Our research group has accumulated a large number of caries images annotated by professional doctors during the preliminary research process. To address the problem of the lack of a digital image dataset of dental caries, we performed data cleaning and image enhancement operations based on the aboveannotated images of dental caries. We deleted the low-quality images in the dataset and further enhanced and expanded the images to build the annotated dataset for dental caries detection. Meanwhile, we here propose use of the RDFNet model (rapid network with deep features for dental caries detection) based on the single-stage deep-learning detection method YOLOv5s to detect dental caries in digital images. Since the caries parts of the images in the dataset are dark and their features are not obvious, RDFNet incorporates the transformer mechanism in the backbone to better extract the complex features of tooth decay and improve the accuracy of detection. To run the caries detection algorithm on portable devices and improve the inference speed, the RDFNet model uses the FReLU activation function to activate the complex visual-spatial information of the images to meet the demand of computing speed.

Overall, the main contributions of this paper are the following.

1. A caries image dataset is constructed, and all images are annotated by professional dentists.
2. The transformer mechanism based on the original YOLOv5 backbone network is incorporated to better extract the complex features of dental caries.
3. The FReLU activation function is adopted to activate the complex visual-spatial information of the images, which improves the inference speed of the model.

## 2. Related Works

### 2.1. Medical Image Object Detection

Object detection is a computer technology related to computer vision and image processing for detecting specific classes of semantic objects (e.g., people, buildings, or cars) in images and videos, which has promising applications in areas such as video security and autonomous driving, among others [6]. Medical images are mainly used to help doctors to make judgments about medical information. Their production has grown exponentially due to the increase of image acquisition devices and advances in camera technology. In recent years, with the continuous development and progress in medical technology, modern hospitals have used medical images to predict the intensity of patients' diseases. Medical object detection based on deep learning has gradually become a current research hotspot. In 2020, Tavakoli et al. [7] used a deep-learning method to detect microaneurysms in retinal images. The experimental results showed that the accuracy of microaneurysm detection was approximately 90%, and the performance of the method using top-hat preprocessing was greater than 80%. During the COVID-19 epidemic, Loey et al. [8] used ResNet50 and YOLOv2 for medical mask-wearing detection. Their proposed model consists of two parts, a deep transfer-learning model based on ResNet50 for feature extraction and a YOLOv2 framework for medical mask detection, achieving a best detection accuracy of 81%.

### 2.2. X-Ray Image-Based Caries Detection

X-ray images are widely used in stomatological research because they show the full details of the teeth and gums. At present, most of the caries detection methods are carried out using X-ray images. Relevant studies have used the method of caries segmentation to detect caries in X-ray images and achieved good accuracy. Rad et al. [9] proposed a caries segmentation and recognition method that uses integral projection technology to extract local feature mapping information of teeth. Lakshmi et al. [10] segmented dental X-ray images using a deep convolutional neural network (CNN) to predict caries in dental images. Both methods demonstrated high accuracy on caries X-ray image datasets. Some studies, such as that of Suryani et al. [2], have also directly used deep-learning methods for caries detection and identification, which saved time and process steps and improved the simplicity of the method.

### 2.3. Transformer

The transformer network is a well-known and efficient deep-learning model proposed by Google in 2017 [11]. The basic version of transformer is based on the attention mechanism and consists of a decoder and encoder. This structure was originally proposed in the sequence-to-sequence model of machine translation [12]. Currently, transformer has been widely used in natural language processing [11], computer vision [13–15], medical disease detection [16], etc. The transformer structure mainly utilizes the self-attention mechanism [11] to extract intrinsic features and has shown great potential in various fields.

Transformer has received significant attention in the field of object detection due to its advantageous capability in extraction of intrinsic features. There are two main categories of transformer-based object detection, a transformer-based set prediction for detection and a transformer-based backbone for detection. DEtection TRansformer (DETR) [13] is a typical example of the first category. A clear disadvantage of this category is the high training cost and poor detection accuracy for small objects. The second type of method takes the transformer structure as a part of the backbone network of common detection methods and has achieved good performance [17].

## 3. Materials and Methods

### 3.1. Dental Caries Annotation Dataset Construction

During preliminary research conducted by our research group, a large number of caries images annotated by professional doctors have been accumulated, but two types of problems exist in the original images. First, there are some low-quality images. The image acquisition equipment contains different models of cameras, smartphones, etc., and the acquired images exhibit large variability in pixels, size, and resolution. Some of the images contain not only the oral part but also the actual living environment of users. Second, some noise exists in the acquired images, and the lighting and contrast in the images are significantly different.

To address the problem of low-quality images in the original data, we conducted data cleaning on the original images, manually selecting and removing unreasonable labels and low-quality pictures one by one according to the annotations in the dataset and only keeping the high-quality images with clear and correct annotations. Then, 7.6% of the original caries images were removed, and a total of 4,277 high-quality caries images were obtained. To address the noise problem in the data, we performed image enhancement operations, e.g., adjusting brightness and contrast, random flipping, and randomly adding noise to the images, to improve the robustness of the model. Specifically, the images in the dataset have been flipped according to 50% probability, and in the process of image flipping, horizontal and vertical flipping were performed separately according to 50% probability. For each image, the brightness, contrast, and saturation were adjusted separately with 33.3% probability. We added noise to the images with 30% probability, and in the process of adding noise, Gaussian, pepper, and salt noise were separately added with 33.3% probability. At the end of all operations, a total of 8,554 images were obtained, including the processed and original images, which realizes the enhancement and expansion of the dataset.

After preprocessing the original data, the labeled dental caries instances were divided into three different categories, i.e., mild, moderate, and severe dental caries according to the clinical manifestations of dental caries at different stages, clinical diagnoses of patients in the hospital, and practical experience of the dentists. The statistics of caries instances for each category are shown in Table 1.

### 3.2. RDFNet

Given the lack of research on digital images for caries detection, the RDFNet model, based on YOLOv5s, which is inspired by the YOLO [18] series algorithm, taking the characteristics of real-time and accuracy into account, is proposed in this study.

The structure of RDFNet is shown in Figure 1. The model contains backbone, neck, and prediction modules.

#### 3.2.1. Overview

The backbone module is used to perform the extraction of caries features. Among them, focus [19] is a slicing operation that can replace convolution and reduce the loss of feature information caused by convolution. C3Modified is a convolution module activated by the FReLU function that is used to extract complex visual-spatial information of caries images. SPP [20] is a spatial feature pyramid pooling structure that can expand the perceptual field, fuse the local and global features, and enrich the information of the feature map. To better extract the depth features of dental caries, RDFNet adds an improved transformer-encoder module after the original SPP structure, which is used to increase the network's ability to extract dental caries features.

The neck module is used to fuse feature maps of different sizes as well as extract high-level semantic features. The module uses the structure of feature pyramid network (FPN [21]) and path aggregation network (PAN [22]), where FPN is performed top-down, the predicted feature maps are obtained by passing fusion of information through upsampling, and PAN is performed bottom-up to obtain the feature pyramids. Feature fusion is performed using top-down as well as bottom-up approaches, thus reducing information loss. To better extract the high-level semantic features of caries images, in this study, the improved C3Modified convolutional module is adopted in the neck module.

The prediction module uses the high-level semantic features generated by the neck module to classify and regress the class and location of objects. It consists of three detection heads to detect large, medium, and small objects, which is a good way to overcome the shortcomings of the single-stage detection method with low detection accuracy for small target objects.

#### 3.2.2. Feature Extraction Module Integrated with Transformer Structure

Since transformer has strong extraction capability for complex features, the feature extraction module shown in Figure 2 is proposed based on transformer's structure.

To extract features better, we perform stacking of three transformer encoders. In our experiments, we remove the original normalization layer from the transformer encoder in order to simplify the model.

We fed the feature map into this structure for the extraction of deep features. The attention values of the different heads were calculated separately and then concatenated. The calculation formulas for calculating the value of multihead attention are

(1) $$\begin{array}{c} \text{MultiHeadAttention}\left(Q,K,V\right)=\text{Concat}\left({\text{head}}_{1},\cdots ,\text{hea}{\text{d}}_{4}\right),\\ {\text{head}}_{\text{i}}=\text{Attention}\left({QW}_{i}^{Q},{KW}_{i}^{K},{VW}_{i}^{V}\right). \end{array}$$

The formula for calculating the value of attention is

(2) $$\begin{array}{c} \text{Attention}\left(Q,K,V\right)=\text{soft}\max\left(\frac{Q\times K^{T}}{\sqrt{d_{k}}}\times V\right), \end{array}$$

where *d*_*k*_ denotes the input dimension, and *Q*, *K*, and *V* denote the query, key, and value matrices, respectively. *Q*, *K*, and *V* in the multihead self-attention mechanism in this modular structure have the same values, which are the values of the input feature maps.

#### 3.2.3. Improved Convolutional Module for Extracting Complex Visual-Spatial Information

Ma et al. [23] identified spatially insensitiveness in activations as the main obstacle impeding visual tasks from achieving significant improvements in vision tasks and proposed a new visual activation function, i.e., FReLU, based on that. Inspired by the ability of FReLU to capture complex visual-spatial information, in the present work, we used the FReLU activation function to improve the original convolution module. The structure of the improved convolution module is shown in Figure 3.

We adopted max(∗) as the nonlinear function and spatial context for each pixel as the condition part. A parametric pooling window was used to create spatial dependency.

(3) $$\begin{array}{c} f\left(x_{c,i,j}\right)=\max\left(x_{c,i,j},T\left(x_{c},i,j\right)\right),\\ T\left(x_{c,i,j}\right)=x_{c,i,j}^{\omega }\;•\;p_{c}^{\omega }. \end{array}$$

Here, *x*_*c*,*i*,*j*_ is the input pixel of the nonlinear activation *f*(·) on the *c* th channel at the two-dimensional spatial position (*i*, *j*). The function *T*(·) denotes the funnel condition, *x*_*c*,*i*,*j*_^*ω*^ a *k*_*h*_ × *k*_*w*_ parametric pooling window centered on *x*_*c*,*i*,*j*_, *p*_*c*_^*ω*^ the coefficient on this window that is shared in the same channel, and (·) dot multiplication.

## 4. Results and Analysis

### 4.1. Experimental Settings

The dataset of digital images constructed in the present work was used in the experiments, with 8,554 caries images divided into training, verification, and test sets according to the ratio of 7 : 2 : 1. The numbers of images in the training, verification, and test sets are 5,987, 1,711, and 856, respectively. To improve the detection accuracy and model robustness, we combined all caries instances in the dataset into one category and detected the caries of this category.

The model was trained using the Pytorch deep-learning framework on an NVIDIA GeForce RTX 3090 graphics card with 24 GB of RAM. The model training parameter settings are shown in Table 2.

### 4.2. Evaluation Criteria

We used three measurements to evaluate the models, namely, accuracy *P*, recall *R*, and average precision mAP@0.5. The calculation formulas are defined as follows:

(4) $$\begin{array}{c} P=\frac{\text{TP}}{\text{TP}+\text{FP}}, \end{array}$$

(5) $$\begin{array}{c} R=\frac{\text{TP}}{\text{TP}+\text{FN}}, \end{array}$$

(6) $$\begin{array}{c} \text{mAP}@0.5=\frac{\sum_{1}^{n}\int_{0}^{1}p\left(r\right)dr}{n}\left(\text{threshold}=0.5\right). \end{array}$$

In formulas (4) and (5) *TP*, *FP*, and *FN* represent true positive, false positive, and false negative, respectively.

In formula (6), *n* denotes the number of classes, *p*(*r*) is the curve between recall and accuracy, and threshold is the Intersection over Union (IoU) threshold of the ground-truth and predicted boxes.

We used frames per second (FPS), i.e., the number of pictures that can be processed per second, as the evaluation criteria of the model detection speed. The calculation formula is defined as follows:

(7) $$\begin{array}{c} \text{FPS}=\frac{\text{frameNum}}{\text{elapsedTime}}, \end{array}$$

where frameNum denotes the total number of pictures that need reasoning, and elapsedTime denotes the total elapsed time of the reasoning process (seconds).

### 4.3. Comparison with Existing Methods

Six deep learning models, i.e., YOLOv5s, YOLOv5m, YOLOv5l, YOLOv3-tiny [24], faster R-CNN [25], and mask R-CNN [26], were used to facilitate separate comparisons with RDFNet, and the experimental results are shown in Table 3. YOLOv5s, YOLOv5m, and YOLOv5l are different improved versions of YOLOv5, and the number of modules and parameters of all three is in the form of incremental increase. YOLOv3-tiny removes some feature layers from YOLOv3 [27] and keeps only two independent prediction branches. Compared with YOLOv3, YOLOv3-tiny has faster computing speed. Faster R-CNN integrates feature extraction, proposal extraction, bounding box regression, and classification in a single network, which has improved the comprehensive performance of the model, especially the detection speed. Mask R-CNN is improved from faster R-CNN by adding a branch of prediction segmentation mask.

As can be seen from the table, the results of the RDFNet method in accuracy and average precision are significantly better than those of the region proposal-based methods, i.e., faster R-CNN and mask R-CNN, but the experimental recall results are the opposite. This is because, at the early stage of dental caries, the difference between lesion and background images is small, and the region proposal-based methods divide the background, etc. into recognition targets when proposing regions, which leads to the reduction of recognition accuracy of the model and to the recall rate deviating from the normal range. Region proposal-based methods take a significant amount of time in proposing regions and thus are slightly inferior to the single-stage object detection methods in terms of recognition speed. However, faster R-CNN effectively improves the speed of proposing regions by using region proposal networks instead of the previous selective search method, resulting in a large improvement in the performance of the model, especially in detection speed, and thus the best detection speed was achieved in the experiments.

In the experiments described herein, YOLOv5s, YOLOv5m, and YOLOv5l did not differ significantly in accuracy, average precision, and recall, but YOLOv5s showed the best results in terms of detection speed. This is because YOLOv5s has a smaller number of parameters compared to YOLOv5m and YOLOv5l; so, the model has a better detection speed overall. Meanwhile, there was no significant difference in other evaluation criteria, indicating that the feature extraction of the model tends to saturate. Because caries in all images are small, this results in limited features extracted by the model, which affects the performance of the method. This situation is not related to the improvement of model complexity and the number of parameters. The detection speed of the RDFNet method is maintained at the same level as in YOLOv5s. This is because the transformer mechanism effectively captures the deeper features in the caries images, while the FReLU activation function accelerates the speed of detection. From the above experimental results, it can be seen that the RDFNet method can effectively improve the accuracy of caries detection while maintaining a fast detection speed, achieving a good balance between accuracy and speed.

### 4.4. Ablation Study

To verify the effectiveness of each part of the model, a series of ablation experiments were designed and conducted; the experimental results are shown in Table 4.

#### 4.4.1. Transformer Mechanism

It can be seen that in the ablation experiments, the accuracy of RDFNet without incorporating the FReLU function was improved by 1.6% compared with RDFNet without incorporating the FReLU function and transformer mechanism. This is because the transformer mechanism extracts deeper features in the image, and these features effectively improve the performance of the model. The accuracy and average precision of RDFNet are improved by 5% and 1.7%, respectively, compared with RDFNet without incorporating the transformer mechanism. The comparison of the results also proves that the transformer mechanism can effectively enhance the model's ability to extract features and improve accuracy.

#### 4.4.2. FReLU Function

RDFNet without incorporating transformer mechanism improved the recall rate by 1.6%, and the detection speed was also improved compared with RDFNet without incorporating the transformer mechanism and FReLU function. This is because the FReLU activation function accelerates the convergence speed of the model and improves its prediction efficiency, while the FReLU activation function can also affect the feature extraction of the model and reduce the missed detection rate. Comparison of the experimental results of RDFNet with and without incorporating the FReLU function show that the RDFNet method alone outperforms the former in all evaluation criteria, which also further verifies the accuracy of the above conclusions.

### 4.5. Comparison of Test Results

To test the caries detection effect of RDFNet, six annotated images were randomly selected in the caries test dataset and compared with the prediction results of the model, arranged according to the real annotated caries images at the top and the prediction results of RDFNet at the bottom. The arrangement is shown in Figure 4.

From the overall view of the six images, the detection result of the six images is satisfying. In Figure 4(a), the lesion area of caries is accurately located. For caries with no obvious characteristics in Figure 4(c) and caries with a small lesion area in Figure 4(e), both instances of caries can still be accurately detected, indicating that RDFNet can effectively detect the caries position in the images.  Figure 4(f) is the image after horizontal flipping; brightness, contrast, and saturation adjustments; and the addition of noise based on the original image. A good detection result is achieved, indicating that RDFNet has good robustness and can cope with more complex application scenarios.

However, errors and omissions are also evident in the test results. In Figures 4(b) and 4(d), some caries in of the image are not detected correctly because they are not particularly obvious compared with other caries, and there is insufficient illumination near caries, which leads to the omission. In Figure 4(e), there is insufficient illumination inside the oral cavity and the inner part of the cavity is dark, resulting in incorrect detection of dental caries by RDFNet.

## 5. Discussion

The objectiveness of this study is to construct a dataset of digital images of dental caries annotated by professional doctors and propose an end-to-end detection method RDFNet for the detection of dental caries.

Therefore, the main contributions of this paper are as follows: a caries dataset annotated by professional dentists was constructed. The RDFNet method is proposed to achieve fast and accurate detection of caries images. In the analysis in the previous section, we can find that the transformer mechanism effectively extracts the feature of dental caries, which is an important reason for RDFNet to prevail. And the FReLU activation function is added to the convolutional module to improve the convergence speed of the model, which makes up for the decrease of the model running speed after the transformer mechanism is added.

The limitation of this study includes that the method does not work well when the internal illumination of oral image is insufficient, and the detection accuracy and speed are improved compared with the original method, but the detection speed is not the fastest among all comparison methods. Hence, future work will concentrate on how to further improve the running speed of the model and improve the performance of the model on images with insufficient illumination.

Since the proposed method has only been validated in an experimental setting, we plan to deploy the model to various devices, including personal computers, smartphones, and embedded devices, in the future. We expect that the method will be applied in subsequent industrial applications and become fundamental for oral care devices, such as smart toothbrushes with caries detection, to promote human dental health.

## 6. Conclusions

Aimed at the problem of a lack of research on caries detection methods based on digital images, we construct a caries image dataset annotated by professional dentists and propose a caries detection method, i.e., RDFNet, according to the requirements of performing caries detection on portable devices. Based on the original YOLOv5s backbone network, this method integrates the transformer mechanism to extract features, improving the detection accuracy. The FReLU activation function is used to activate the complex visual-spatial information of the image, which accelerates the reasoning speed of the model. RDFNet method can effectively improve the accuracy of caries detection while maintaining a fast detection speed at the same time. In the future, the RDFNet method will be applied to various devices for dental caries detection and promote human dental health.

## Figures and Tables

**Figure 1:** RDFNet structure.

**Figure 2:** Feature extraction module integrated with transformer structure.

**Figure 3:** Improved convolution module structure.

**Figure 4:** Comparison of real annotated caries images and predicted results using the proposed method.

**Table 1:** Statistics of caries instances in the dataset constructed in the present work.

Categories	Total number	Percentage
Mild caries	5,570	38.1%
Moderate caries	4,370	29.9%
Severe dental caries	4,670	32.0%

**Table 2:** Training parameter settings for proposed method.

Parameter	Value	Parameter	Value
Input size	640	Epoch	80
Initial learning rate	0.001	Decay	0.0005
Momentum	0.937	Batch size	32
Optimizer	Steepest gradient descent	Multiscale training	False

**Table 3:** Comparison between RDFNet and other object detection methods. The italic value indicates the top performance.

Methods	*P*	mAP@0.5	*R*	FPS
YOLOv5s	0.597	0.552	0.578	20.12
YOLOv5m	0.608	0.556	0.585	18.94
YOLOv5l	0.606	0.563	0.582	17.98
YOLOv3-tiny	0.589	0.5	0.566	22.74
Faster R-CNN	0.421	0.421	*0.825*	*23.14*
Mask R-CNN	0.42	0.42	0.824	17.89
RDFNet	*0.623*	*0.569*	0.579	20.24

**Table 4:** Results of RDFNet ablation experiments. The italic value indicates the top performance, and “w/o” indicates “without.”

Methods	*P*	mAP@0.5	*R*	FPS
RDFNet w/o transformer and FReLU	0.597	0.552	0.578	20.12
RDFNet w/o FReLU	0.613	0.554	0.578	20.19
RDFNet w/o transformer	0.573	0.552	*0.604*	*20.56*
RDFNet	*0.623*	*0.569*	0.579	20.24

## Data Availability

Considering the privacy of patients, we cannot open access to our clinical data.
